# Activating Transcription Factor 3 Based Early Alarm Model of Acute Kidney Injury after Cardiopulmonary Bypass in Adults

**DOI:** 10.1155/2022/8076718

**Published:** 2022-10-11

**Authors:** Xiao-Yun Wu, Xiang-Lan Jin, Qiang Liu, Feng Qiu, Jian Zhou

**Affiliations:** Department of Cardiac Surgery, Shanghai Tenth People's Hospital, School of Medicine, Tongji University, Shanghai 200072, China

## Abstract

Acute kidney injury (AKI) is a common complication after cardiopulmonary bypass (CPB) for cardiac surgery, and there is no effective treatment. This study was aimed at constructing an early warning model of AKI after CPB in adults and investigating the performance of this model. Patients who underwent CPB in the Department of Cardiac Surgery, Shanghai Tenth People's Hospital, from January 2018 to December 2019 were recruited into the present study. Blood and urine samples were collected preoperatively (0 h) and 2 h, 6 h, 12 h, 24 h, and 48 h after surgery, and the creatinine and activating transcription factor 3 (ATF3) were detected. According to the diagnostic criteria of AKI, patients were divided into the AKI group and the non-AKI group, and the risk factors for AKI after CPB were screened. The receiver operating characteristic (ROC) curve analysis was used to identify the optimal biomarkers for the establishment of early warning model of AKI after CPB. Finally, the performance of this model was further verified. A total of 83 patients were included in this study, 42 of whom developed AKI after surgery. After CPB, the serum and urine levels of creatinine and ATF3 increased to different degrees, and the increase in urine ATF3 was the most obvious in the AKI group. The area under ROC (AUC) of urine ATF3 at 12 h after surgery was 0.691 (95% CI: 0.576-0.807). When ATF3 was higher than 1216 pg/mL, the sensitivity and specificity of ATF3 in the diagnosis of AKI were 0.43 and 0.85, respectively. The height, conjugated bilirubin on the surgery day, urine ATF3 12 h after surgery, and serum creatinine 24 h after surgery were independent risk factors for postoperative AKI. Urine ATF3 and other factors were used to establish AKI warning model after CPB, which showed good fitting and accuracy. In conclusion, ATF3 is an early biomarker of post-CPB AKI. Addition of urine ATF3 to AKI risk factors can improve the accuracy of early AKI prediction.

## 1. Introduction

Acute kidney injury (AKI) is one of the most common complications after major surgery, especially after cardiac surgery [1, 2]. Despite significant improvements in perioperative management, the incidence of AKI in the intensive care units (ICU) remains high, ranging from 20% to 67% [3]. Currently, there is no effective treatment for AKI, and studies have focused on the early detection, diagnosis, and prevention of AKI after surgery. To date, many biomarkers have been identified for the early diagnosis of AKI, but their sensitivity and specificity are still low. Therefore, establishing early warning model for AKI and identifying patients at high risk of AKI after cardiac surgery are crucial to prevent the postoperative AKI.

Studies have shown that activating transcription factor 3 (ATF3) is detectable in the urine within 2-24 h in the rat AKI model [4]. Panich et al. [5] found a similar pattern of urinary ATF3 in patients with sepsis-induced AKI. Our previous study suggested that ATF3 could be expressed early in patients with AKI after cardiac surgery [6]. This study was aimed at investigating whether ATF3 could serve as a risk variable and at establishing an early alarm model for AKI in patients receiving cardiopulmonary bypass (CPB) heart surgery.

## 2. Materials and Methods

This study was registered in the Chinese Clinical Trial Registry (ChiCTR2000030869) and approved by the Ethics Committee of Shanghai Tenth People's Hospital (2019-K-20). Patients who underwent CPB in the Department of Cardiac Surgery, Shanghai Tenth People's Hospital, from January 2018 to December 2019 were recruited into present study. The inclusion criteria were as follows: (1) all patients underwent elective CPB; (2) patients were older than 18 years but younger than 80 years; (3) informed consent was obtained from each patient prior to the study; and (4) patients were conscious and able to cooperate with the clinicians. The exclusion criteria were as follows: (1) the expected hospital stay was no more than 3 days; (2) patients had a history of chronic kidney disease; (3) preoperative vital signs were unstable; (4) patients developed urinary tract infection within 3 days before surgery; and (5) there was a critical condition after CPB.

### 2.1. Methods

#### 2.1.1. Collection of Clinical Information

With “Cardiac surgery,” “Cardiopulmonary bypass/CPB,” “acute kidney injury/AKI,” and “risk factor” as terms, the main databases (PubMed, Ovid, and Medline) were searched for related studies. The retrieved studies were reviewed and summarized, and the identified risk factors were included into this study and divided into preoperative, intraoperative, and postoperative ones. These factors included gender, age, height, weight, left ventricular ejection fraction (LVEF), hypertension, diabetes mellitus, findings from preoperative routine blood test, findings from preoperative liver and kidney function detection, name of surgery, duration of CPB, duration of aortic occlusion, intraoperative blood transfusion, ICU stay, duration of mechanical ventilation, findings from routine blood test on the operation day, findings from the liver, and kidney function detection on the operation day, use of vasoactive drug, complications, and outcomes.

#### 2.1.2. Collection, Processing, and Storage of Samples

The blood and urine samples (3 mL for each) were collected before surgery (0 h) and 2 h, 6 h, 12 h, 24 h, and 48 h after surgery. All samples were centrifuged, and the supernatant was collected, transferred into an Eppendorf tube, and stored at -80°C. Blood and urine ATF3 was detected with corresponding ELISA kit (human ATF3 kit, 96 Tests, CloudClone Crop). Additionally, blood and urinary creatinine (Cr) was detected in the Department of Laboratory.

#### 2.1.3. Grouping

According to the diagnostic criteria for AKI recommended by the Kidney Disease: Improving Global Outcomes (KDIGO), patients were divided into the AKI group and non-AKI group, and the renal function and urine and blood ATF3 levels were compared between two groups at different time points. Specifically, the definition of AKI is as follows: renal function deteriorates rapidly within 48 h after surgery, the absolute serum Cr rises ≥26.5 *μ*mol/L (0.3 mg/dL) or ≥1.5 times the baseline level, or the urine volume is <0.5 mL/kg/h for 6 h. The baseline serum Cr level referred to the value on admission.

### 2.2. Statistical Analysis

Statistical analysis was performed with Statistical Product and Service Solutions (SPSS) version 19.0 (SPSS Inc., Chicago, IL, USA). Quantitative data with normal distribution were expressed as the mean ± standard deviation (SD) and compared with a *t*-test; quantitative data without normal distribution were expressed as median (lower interquartile, upper interquartile) and compared with the Wilcoxon test. Qualitative data were compared with a chi-square test or the Fisher exact test. Repeated measures analysis of variance was used to compare the biological markers at different time points in two groups. At last, the receiver operating characteristics (ROC) and area under the ROC curve (AUC) were employed to evaluate the performance of ATF3, in the diagnosis of AKI.

The patients' characteristics at baseline were subjected to univariate analysis, and factors with *P* < 0.15 were included for further multivariate logistic regression analysis. The logistic regression analysis was used to establish the model in which the factors with *P* < 0.2 in the univariate analysis were included; stepwise regression analysis was done for the screening of factors (inclusion: *α* = 0.05; exclusion: *α* = 0.1), and an early alarm model was established for AKI. After resampling with the Bootstrap method, internal cross-validation was performed (1000 times); the calibration curve, Hosmer and Lemeshow goodness of fit test, Intercept, Slope, *C*-index, Brier scaled, and *R*^2^ were used for the assessment of this model. The accuracy of this model was evaluated by Bootstrap verification and calibration verification (Figure 1).

## 3. Results

### 3.1. Clinical Characteristics at Baseline, Surgeries, and Outcomes

A total of 83 patients with an average age of 60.47 ± 10.47 years were recruited into this study, including 48 males (57.83%) and 35 females (42.17%). Of these patients, 34 had coronary artery bypass graft surgery, 3 had coronary artery bypass graft surgery plus valve surgery, 39 had valve surgery (single or dual valve replacement), 2 had large vessel surgery, and 5 had other procedures (surgery for tumors, atrial fibrillation ablation, repair of atrial septal defects, etc.).

All patients underwent cardiac surgery successfully, with a mean ICU stay of 74.78 ± 65.07 h and a mean ventilation time of 27.64 ± 58.61 h. Three patients died after surgery due to postoperative sepsis, multiple organ failure, and sudden cardiac death within 1 week, and two patients received continuous renal replacement therapy.

### 3.2. Incidence of AKI and Univariate Analysis

AKI was found in 42 patients (50.6%), including 20 males (47.62%) and 22 females (52.38%). The average age was 62.76 ± 10.18 years. There were 7 patients with diabetes mellitus (16.67%) and 21 patients with hypertension (51.22%). The preoperative LVEF and the serum Cr were 58.48 ± 8.50 mL and 75.07 ± 17.71 *μ*mol/L, respectively.

Univariate analysis showed significant differences in the age, height, preoperative hemoglobin, alanine aminotransferase, and blood urea nitrogen between the AKI group and the non-AKI group. Significant differences were observed in the platelet and blood urea nitrogen on the day of operation between two groups (*P* < 0.05). However, other baseline characteristics, comorbidities, baseline cardiac function, duration of CPB, ICU stay, duration of mechanical ventilation, and postoperative complications were comparable between two groups (Supplementary Table 1).

### 3.3. Perioperative Serum and Urine Levels of Creatinine and ATF3

The serum Cr was significantly higher in the AKI group at 12 h postoperatively (102.57 *μ*mol/L *vs.* 73.21 *μ*mol/L) than in the non-AKI group, but the diagnosis of AKI required the examination 24 h postoperatively according to the diagnostic criteria for AKI (the absolute serum Cr rises ≥26.5 *μ*mol/L from the baseline). The urine Cr level in the AKI group peaked at 12 h after surgery (5.44 mmol/L), but there was no significant difference between the AKI group and non-AKI group (Table 1).

Serum ATF3 at 24 h after surgery in the AKI group was significantly higher than in the non-AKI group (662.62 ± 204.72 pg/mL *vs*.586.93 ± 175.87 pg/mL, *P* = 0.04). However, the urine ATF3 in the AKI group was markedly higher than in the non-AKI group at 6 h postoperatively (974.92 ± 341.42 pg/mL *vs* 1169.90 ± 280.93 pg/mL, *P* = 0.01), and this significant difference was also observed at 12 h postoperatively (993.23 ± 291.16 pg/mL *vs* 1190.05 ± 309.58 pg/mL, *P* = 0.002) (Table 1).

Repeated measures analysis of variance showed that the variation of each biological marker was different at different time points (*P* < 0.05); however, only serum Cr and urine ATF3 showed differences in different groups. After analysis of the interaction between time and groups, serum Cr, blood, and urine ATF3 had better significance (*P* < 0.001, *P* = 0.02, and *P* = 0.008, respectively) (Table 2).

### 3.4. Role of Serum ATF3 in the Diagnosis of AKI

As shown in Table 3, serum Cr, a gold standard for the diagnosis of AKI at present, displayed obvious advantages in the ROC analysis. The AUC of urine ATF3 at 12 h after surgery was the largest, and thus, it could be used as a diagnostic marker for AKI (AUC = 0.691; 95% CI 0.576-0.807; sensitivity: 0.43; specificity: 0.85).

### 3.5. Determination of Risk Factors

The preoperative characteristics of patients (including height, weight, gender, age, eGFR, LVEF, and various preoperative examinations), surgery-related information, findings from examinations on the day of surgery, perioperative Cr, and ATF3 served as variables. Then, the independent risk factors of post-operative AKI were screened using a backward method with a *P* value threshold of 0.05 (Table 4).

### 3.6. Establishment of Model

After multivariate logistic analysis, the risk factors for postoperative AKI were employed to establish the prediction model of postoperative AKI. The regression equation was as follows:

Logistic regression equation:

(1) $$\begin{array}{c} P=\frac{\exp\left(\beta_{0}+\beta_{1}X_{1}+\beta_{2}X_{2}+\beta_{3}X_{3}+\cdots +\beta mXm\right)}{1+\exp\left(\beta_{0}+\beta_{1}X_{1}+\beta_{2}X_{2}+\beta_{3}X_{3}+\cdots +\beta mXm\right)}. \end{array}$$

### 3.7. Verification of Model

After resampling with the Bootstrap method, the internal cross-validation was performed. Calibration curve, Hosmer and Lemeshow GOF test, Intercept, Slope, *C*-index, Brier scaled, and *R*^2^ were used for the assessment of this model. For this model, the Intercept was -0.0018, the Slope was 0.7177, the *C*-index (ROC) was 0.9181, the Brier scaled was 0.1315, and the *R*^2^ was 0.6501. The GOF test showed the *X*-squared was 10.666, and the *P* value was 0.2213. These suggested good fitting of this model (Figure 2).

### 3.8. The Model and ROC Analysis

The established model was displayed as the Nomograms. When the total Nomogram score of 119.22 served as a cut-off value, the AUC was 0.9409 with the sensitivity of 85.71%, specificity of 89.66%, positive predictive value of 89.29%, and negative predictive value of 87.10% (Figures 3 and 4).

## 4. Discussion

AKI refers to the abrupt decrease in the renal function. It is a common and serious complication in adults after CPB and has high morbidity and mortality [1, 2, 7–10]. Its incidence was 31% in the study by Leon et al. [2] and was as high as 59% in the study by Kwiatkowski et al. [7]. AKI after cardiac surgery not only affects the prognosis of patients but also increases the in-hospital and postdischarge mortality of patients. Studies have demonstrated that [8] the in-hospital mortality of AKI patients after CPB is 7.3-50%. Hirano et al. [9] conducted a long-term follow-up of patients with AKI after CPB and found that the occurrence of AKI would increase the mortality two years after surgery.

Currently, there are no widely acceptable biomarkers for the diagnosis of AKI. Many biomarkers have been identified for the diagnosis and prediction of AKI, but many of them have lower sensitivity and lower specificity (<70%-75%) [10]. For example, the determination of Cystatin C (CysC) in patients with proteinuria is affected due to blocked reabsorption [11]. Also, the detection of neutrophil gelatinase-associated lipocalin will be affected in some cases of prerenal diseases, systemic or urinary system infections, resulting in bias in the results [12]. Thus, to establish an early alarm model of AKI has become crucial to prevent the occurrence and deterioration of AKI and to reduce the mortality.

Most existing models preoperatively predict AKI risk based on the baseline characteristics of patients [13, 14], while some models have an end point of AKI treated with renal replacement therapy [15, 16, 17]. The Cleveland Clinical Score [15], developed by Thakar et al., is the most widely used risk prediction model for AKI after cardiac surgery currently [13]; however, in the external validation of this model, results are not satisfactory [18]. Therefore, researchers have proposed that the introduction of new AKI biomarkers may change the current diagnostic criteria for AKI and improve the predictive performance of these models [19].

Our study proved that ATF3, one of members of the ATF/CREB subfamily of the basic Leucine zipper family, was also a good biomarker for AKI, which is consistent with previous findings [4, 5]. To be specific, in patients with AKI after CPB, the urine and serum ATF3 levels increased, especially urine ATF3 (*P* < 0.05). The significant increase in the urine ATF3 occurred earlier than in the serum ATF3 (12 h *vs.* 24 h after surgery). The urine ATF3 at 12 h after surgery was >1216 pg/mL, and its AUC was 0.691 (95% CI 0.576-0.807) with the sensitivity of 0.43 and specificity of 0.85 in the diagnosis of AKI, which was better than that of serum ATF3 and urine ATF3 at other time points. In addition, there was interaction between time and groups in the urine ATF3. Therefore, we speculate that ATF3 can be used as a new and effective marker for predicting AKI, especially for the patients receiving heart surgery.

In order to identify the risk factors of post-operative AKI, all the perioperative biological markers were included in the variable screening of the model, in addition to the baseline perioperative clinical characteristics. According to the analysis results, height, bilirubin level on the day of surgery, urinary ATF3 at 12 h after surgery, and serum Cr at 24 h after surgery were independent risk factors for AKI, but eGFR, LVEF, operation time, and reoperation were not identified as risk factors as in previous studies. In addition, our results also showed that urine ATF3 was an independent risk factor, which confirmed the possibility of ATF3 as a predicting marker for AKI.

Although there were few risk factors included, the internal cross-validation of the model showed satisfactory; the estimated incidence of AKI was basically consistent with the actual incidence by the model, indicating good fitting (Figure 2). The model converted into a Nomogram score table was more convenient and intuitive to use in clinical practice (Figure 3). Based on each patient's data, the corresponding value can be found on the score sheet and the total score can be calculated. If the cut-off value of Nomogram score was 119.22, the AUC of this model was 0.9409 with the sensitivity of 85.71%, the specificity of 89.66%, the positive predictive value of 89.29%, and the negative predictive value of 87.10% in the diagnosis of AKI (Figure 3). Its AUC was higher than that reported in previous studies [13–17, 20–25]. Thus, our model is promising to be used as a tool to identify high-risk patients clinically.

The early alarm model of AKI after CPB in this study was internally validated to have high accuracy and practicability, and it may provide clinicians with a new and effective tool to identify the AKI risk in the future. However, there are still several limitations in this study. First, the sample size was still small, and only 83 patients were included. Therefore, more studies with large sample size are needed to confirm our findings. Second, the endpoint of this retrospective study was the occurrence of AKI. Most patients had stage 1 or stage 2 AKI, and there was no AKI requiring renal replacement therapy in the present study, which may increase the difficulty in the risk factor screening. Third, only internal validation of the original data was done in this model, and external validation was not performed with large sample size. Forth, our model was established based on the clinical characteristics of patients receiving CPB for cardiac surgery, but whether this model is also applicable in patients receiving other types of cardiac surgery is still unclear.

## 5. Conclusion

AKI is a common and serious complication after CPB for cardiac surgery, and early diagnosis can improve its clinical outcomes. Our study shows ATF3 can be a biomarker for early predicting AKI after CPB, and the addition of urine ATF3 as a risk factor to the AKI alarm model can improve the accuracy of early prediction of AKI.

## Figures and Tables

**Figure 1:** Study flow chart.

**Figure 2:** Calibration curves. *X*-axis: predicted rate of the model; *Y*-axis: actual rate of AKI. Apparent represents the estimated curve of the model; Bias-correct is a curve after cross-validation. Cross-validation was done by 1000 repetition of Bootstrap analysis. According to the calibration curves, the Apparent and Bias-correct curves of this model overlapped with the ideal curve, suggesting a good fit of the model.

**Figure 3:** Nomogram analysis of model. The value of each variate was input into a table, and each variate was scored based on their absolute value. The sum of scores of each factor was calculated; the higher the score, the higher the risk for postoperative AKI.

**Figure 4:** ROC analysis of the model. When the Nomogram score was larger than 119.22, the AUC of this model was 0.9409 with the sensitivity of 0.8571, specificity of 0.8966, positive predictive value (PPV) of 0.8929, and negative predictive value (NPV) of 0.8710 in the diagnosis of AKI.

**Table 1:** Perioperative urine and blood creatinine and ATF3 in two groups.

Variables	0 h	2 h	6 h	12 h	24 h	48 h
Serum Cr (mmol/L)						
Non-AKI	76.82 ± 18.45	75.42 ± 19.05	65.11 ± 19.87	65.08 ± 23.85	79.12 ± 19.06	77.52 ± 21.61
AKI	73.21 ± 17.64	81.04 ± 20.30	85.85 ± 45.48	88.65 ± 29.23	102.57 ± 28.51	105.06 ± 35.47
T	0.94	-1.56	-2.82	-3.89	-4.35	-4.27
P	0.35	0.12	0.006	<0.001	<0.001	<0.001
Urine Cr (mmol/L)						
Non-AKI	3.74 ± 2.42	3.79 ± 2.35	3.71 ± 2.23	4.67 ± 2.22	4.56 ± 2.68	5.23 ± 2.35
AKI	3.73 ± 2.62	3.91 ± 2.54	5.29 ± 5.91	5.44 ± 2.85	4.85 ± 2.39	4.02 ± 2.38
T	-0.12	0.22	-1.61	-1.62	-1.25	2.17
P	0.90	0.83	0.11	0.11	0.21	0.03
Serum AATF3 (pg/mL)						
Non-AKI	530.12 ± 155.97	628.12 ± 202.44	710.87 ± 197.43	753.97 ± 216.57	586.93 ± 175.87	503.29 ± 146.32
AKI	489.18 ± 134.00	596.67 ± 159.23	759.86 ± 188.87	774.96 ± 203.22	662.62 ± 204.72	518.22 ± 130.62
T	0.94	0.90	-1.47	-0.92	-2.15	-0.54
P	0.35	0.54	0.14	0.36	0.03	0.59
Urine ATF3 (pg/mL)						
Non-AKI	746.99 ± 255.36	868.98 ± 212.99	974.92 ± 341.42	993.23 ± 291.16	839.52 ± 308.14	728.70 ± 212.39
AKI	733.30 ± 175.79	924.74 ± 217.65	1169.90280.93	1190.05 ± 309.58	924.15 ± 253.07	780.55 ± 277.70
T	0.29	-0.95	-2.53	-3.14	-1.52	-1.07
P	0.77	0.34	0.01	0.002	0.13	0.29

**Table 2:** Repeated measures ANOVA for creatinine and ATF3.

Variables		Time	Time × group	Group
Serum Cr (*μ*mol/L)	*F*	10.54	6.83	15.54
	*P*	<0.0001	<0.0001	0.0002

Urine Cr (mmol/L)	*F*	2.41	1.93	0.36
	*P*	0.04	0.09	0.55

Serum ATF3 (pg/mL)	*F*	62.02	2.71	0.17
	*P*	<0.0001	0.02	0.68

Urine ATF3 (pg/mL)	*F*	40.46	3.19	3.94
	*P*	<0.0001	0.008	0.05

Notes: “Time” is the main effect of Time. “Group” is the main effect of a Group. “Time × Group” represents the interaction between time and groups.

**Table 3:** ROC analysis of creatinine and ATF3.

	Cut-off	AUC (95% CI)	Sensitivity	Specificity
Serum Cr				
2 h	71.30	0.602 (0.48-0.73)	0.64	0.51
6 h	89.00	0.665 (0.55-0.78)	0.33	0.90
12 h	74.00	0.729 (0.61-0.84)	0.69	0.68
24 h	97.90	0.740 (0.63-0.84)	0.52	0.82
48 h	78.60	0.748 (0.64-0.85)	0.73	0.65
Serum ATF3				
2 h	549.00	0.522 (0.39-0.65)	0.50	0.41
6 h	680.64	0.623 (0.50-0.74)	0.62	0.63
12 h	840.24	0.571 (0.44-0.70)	0.40	0.78
24 h	643.00	0.647 (0.52-0.77)	0.43	0.80
48 h	513.00	0.567 (0.43-0.70)	0.40	0.78
Urine Cr				
2 h	2.11	0.521 (0.39-0.65)	0.59	0.22
6 h	3.68	0.606 (0.41-0.73)	0.59	0.58
12 h	5.41	0.590 (0.40-0.70)	0.57	0.65
24 h	3.92	0.580 (0.45-0.71)	0.64	0.54
48 h	4.87	0.672 (0.53-0.81)	0.16	0.56
UrineATF3				
2 h	843.00	0.548 (0.42-0.67)	0.60	0.54
6 h	1055.84	0.666 (0.55-0.78)	0.62	0.71
12 h	1216.00	0.691 (0.57-0.80	0.43	0.85
24 h	770.02	0.61 (0.49-0.74)	0.64	0.54
48 h	865.48	0.57 (0.43-0.71)	0.26	0.85

**Table 4:** Independent risk factors of postoperative AKI.

Variables	*β*	OR (95% CI)	*P*	*C*-index
Screening				0.9409
Height	-0.227	0.797 (0.689-0.921)	0.002	
Conjugated bilirubin on the day of surgery	2.348	10.459 (1.228-89.076)	0.032	
Serum Cr at 24 h	0.117	1.125 (1.050-1.205)	<0.001	
Urine ATF3 at 12 h	0.006	1.006 (1.002-1.010)	0.003	

## Data Availability

The data used to support the findings of this study are available from the corresponding author upon request.

## Supplementary Materials

Supplementary Materials Supplementary Table 1: patients' characteristics at baseline.
